The article "Effects of Growth Hormone Replacement on Peripheral Muscle and Exercise Capacity in Severe Growth Hormone Deficiency" was published in 2018. Journal: Front Endocrinol (Lausanne).

# Effects of Growth Hormone Replacement on Peripheral Muscle and Exercise Capacity in Severe Growth Hormone Deficiency

**DOI:** 10.3389/fendo.2018.00056

**Published:** 2018-02-23

**Authors:** Susana Gonzalez, Thozhukat Sathyapalan, Zeeshan Javed, Stephen L. Atkin

**Affiliations:** ^1^Hull York Medical School, University of Hull, Heslington, United Kingdom; ^2^Weill Cornell Medicine Qatar, Doha, Qatar

**Keywords:** GH deficiency, succinate dehydrogenase, cardiovascular risk factors, exercise performance, mitochondrial dysfunction

## Abstract

**Objective:**

The aim of this study is to evaluate the effect of growth hormone therapy (rGH) on mitochondrial function on peripheral muscle and to correlate with exercise capacity in subjects with severe adult growth hormone deficiency (GHD).

**Design:**

Six months, double-blind, randomized, crossover, placebo-controlled trial of subcutaneous rGH in 17 patients with GHD.

**Measurements:**

Quadriceps muscle biopsies were obtained at baseline, 3 months, and 6 months to measure succinate dehydrogenase (SDH) to assess mitochondrial activity. Exercise capacity was measured with cardiopulmonary exercise testing. Lipids, glycemic parameters, and body fat levels were also measured.

**Results:**

Serum insulin-like growth factor 1 (IGF1) levels reduced fat mass by 3.2% (*p* < 0.05) and normalized with rGH in the active phase (*p* < 0.005). Patients showed an increase in SDH (*p* < 0.01) from base line that differed between placebo and rGH therapy treatment groups (*p* < 0.05): those treated by rGH followed by placebo showed a significant increase in SDH (*p* < 0.001) followed by a decrease, with a significant between group difference at the end of 6 months (*p* < 0.05). No significant improvements or correlation with exercise capacity was found.

**Conclusion:**

Short-term rGH for 3 months normalized IGF1 levels, reduced fat mass, and had a significant effect on mitochondrial function, but exercise capacity was unchanged.

**Clinical Trial Registration:**

Number ISRCTN94165486.

## Introduction

Patients with hypopituitarism have reduced life expectancy when compared to the general population, mainly attributed to cerebrovascular and cardiovascular disease (1, 2). The cause of this is unclear but induced mitochondrial dysfunction due to increased oxidized LDL, hypertriglyceridemia, and hyperglycemia seen in growth hormone deficiency (GHD) may trigger an increase in mitochondrial reactive oxygen species (ROS) and superoxide molecules formation. The electron transport chain found in the mitochondria is a major site of ROS generation, mainly in the membrane-bound complexes I and III, playing an important role in signaling pathways required for the skeletal muscle adaptation (3). Succinate dehydrogenase (SDH) or respiratory complex II is a crucial antioxidant enzyme also located in the inner mitochondrial membrane and is the only enzyme that participates both in the electron transport chain and in the citric acid cycle. SDH deficiency is associated with mitochondrial disorders that mainly affect organ dependant on oxidative metabolism such as brain, skeletal muscle, and cardiac muscle (4), and it is sensitive to inhibition by ROS complexes (5). Potentially this mitochondrial dysfunction may decrease aerobic capacity and endothelial dysfunction/apoptosis (5).

The article "Effects of Growth Hormone Replacement on Peripheral Muscle and Exercise Capacity in Severe Growth Hormone Deficiency" was published in 2018. Journal: Front Endocrinol (Lausanne).

Diminished aerobic capacity has been identified as an additional independent risk factor for all-cause and cardiovascular mortality in healthy subjects without documented coronary artery disease (6). Maximal oxygen uptake (VO_2_ max) is widely accepted as the single best measure of cardiovascular fitness and maximal aerobic power and represents the maximum capacity of an individual’s body to use oxygen during incremental exercise. Studies assessing VO_2_max in GHD have reported a reduction in aerobic capacity associated with a decreased VO_2_max up to 28% (7, 8) when compared with predicted values (9), indicating reduced cardiovascular fitness. Therefore, measures of aerobic performance could be used to objectively assess the functional response following GH replacement.

Several hormones including thyroid, sex steroids, glucocorticoids, and GH influence skeletal muscle growth and function. The growth-promoting effects of GH are mainly mediated by serum insulin-like growth factor 1 (IGF1); however, available evidence also suggests a GH-independent IGF1 effect as the growth response is better when GH-deficient patients are treated with GH in comparison to IGF1 treatment in patients with GH insensitivity (10).

GH binding to its receptors modulate its effects in the mitochondria (11, 12) through which GH may increase mitochondrial oxidative capacity in the cardiac and skeletal muscle. This was suggested in studies in healthy subjects who received a GH infusion for 14 days (13) and in older women when it was combined with aerobic exercise (14); therefore, this could theoretically be a mechanism by which GH replacement could improve muscle function in patients with GHD. GH stimulates the synthesis of IGF1 in most tissues, and although circulating IGF1 is mainly secreted by the liver in response to GH action, locally synthesized IGF1 isoforms may have an autocrine or paracrine function in the skeletal muscle (10, 15). Higher levels of ROS have also been reported to downregulate IGF1 signaling potentially inducing insulin resistance (16).

The article "Effects of Growth Hormone Replacement on Peripheral Muscle and Exercise Capacity in Severe Growth Hormone Deficiency" was published in 2018. Journal: Front Endocrinol (Lausanne).

To date, it is unknown if GHD is associated with muscle mitochondrial dysfunction. Therefore, the aim of this study is to evaluate the effects of short term administration of GH on peripheral muscle oxidative capacity using SDH activity as a surrogate marker and whether this correlated with exercise capacity and cardiovascular risk markers.

## Subjects and Methods

Seventeen patients (10 males and 7 females; mean age, 48 ± 14 years) with hypopituitarism resulting from pituitary tumors who were treated with surgery, radiotherapy, or both were recruited. Severe GHD was confirmed by a peak GH response to insulin-induced hypoglycemia of less than 9 mU/L (3 ng/mL). The average time from diagnosis of the pituitary lesion to inclusion in the trial was 33 months with confirmation of severe GHD 12 months prior to inclusion in the trial. Subjects were on stable hormone replacement doses for thyroid, adrenal, and testosterone deficiencies for the previous 6 months prior to the study and throughout the study, and no adjustment of the doses were needed during the study. None of them had been previously treated with rGH (Table 1). During the study period, they were instructed to follow their usual diet and activity. All subjects provided written consent.

**Table 1:** Patient demographics.

Patient	Sex	Age	Diagnosis	Time from diagnosis to entry into trial (months)	Therapy
1	M	51	Post Sx: pituitary macroadenoma	15	–
2	M	64	Post Sx: microprolactinoma	13	A
3	F	48	Post Sx: pituitary macroadenoma	22	A, B
4	M	46	Post Sx: pituitary macroadenoma	23	A, E
5	F	54	Post Sx: pituitary macroadenoma	9	A, B
6	F	28	Post Sx: pituitary macroadenoma	3	B
7	F	19	Cystic prolactinoma	19	C
8	M	50	Post Sx: acromegaly	25	–
9	F	58	Post Sx: pituitary macroadenoma	40	B
10	F	36	Post Sx: prolactinoma	2	B
11	M	30	Post Sx: craniopharyngioma	27	A, B
12	F	44	Empty sella	20	C
13	M	44	Post Sx: prolactinoma	27	A, D, E
14	M	69	Post Sx and RTX: pituitary adenoma	45	A, B, E
15	M	62	Post Sx: pituitary macroadenoma	22	A, E
16	M	49	Post Sx: pituitary macroadenoma	68	A, B, E
17	M	64	Post Sx: pituitary macroadenoma	18	–

*A, thyroxine 125 μg daily; B, hydrocortisone (25 mg daily); C, quinagolide (75 μg daily); D, cabergoline (0.5 mg twice weekly); E, Sustanon (250 mg thrice weekly); Sx, surgery*.

This was a 6-month, double-blind, randomized, crossover, placebo-controlled trial of subcutaneous recombinant GH (Lilly rGH^®^, 0.4 mg/day for 12 weeks) versus placebo (sterile diluent containing glycerol and m-cresol, for 12 weeks). The patients were randomized with a random generator table and, using a crossover design, allocated to study group A or B. Daily rGH or placebo injections were prepared by a pharmacist, which was separate from the trial. Nine patients in one arm and eight in the second arm were randomized to either placebo or rGH for 3 months before being crossed over to the second arm of the study following a 2-week washout period for a further 3-month period (Figure 1). To maintain the blinding of the study, it was not possible to escalate the GH dose. Compliance was monitored based on counting the returned empty vials of the study medication.

The article "Effects of Growth Hormone Replacement on Peripheral Muscle and Exercise Capacity in Severe Growth Hormone Deficiency" was published in 2018. Journal: Front Endocrinol (Lausanne).

**Figure 1:** Flow chart describing the progress of patients through the trial.

The study followed the declaration of Helsinki guidelines and was approved by the Hull and East Riding ethics committee. The trial registration number is ISRCTN94165486.

### Study Measurements

At the beginning and end of each phase, following an overnight fast, weight and blood pressure were measured, and blood samples were collected. Blood pressure was measured after the patients had been seated quietly for at least 5 min with the right arm supported at heart level. Blood pressure measurements were performed using an automated device (NPB-3900; Nellcor Puritan Bennett, Pleasanton, CA, USA) during each study visit. Two readings were obtained at the beginning of each visit at least 1 min apart, and the mean value was taken. Total body fat was measured with the bioelectrical impedance analysis technique using Tanita scales (Tanita, IL, USA). Fasting venous blood samples were collected, separated by centrifugation at 2,000 *g* for 15 min at 4°C, and the aliquots stored at −80°C within 1 h of collection. Plasma glucose was measured using a Synchron DxC analyzer (Beckman-Coulter, UK), and total cholesterol, triglycerides, and high-density lipoprotein cholesterol levels were measured enzymatically using a Synchron LX20 analyzer (Beckman-Coulter, UK). IGF1 was measured using a solid-phase, enzyme-labeled chemiluminescent immunocentric assay on an Immulite 2000 analytical platform (Siemens/DPC, DPC-UK, Llanberis, Caernarfon, UK.). IGF1 SDS measurements were calculated from the online calculator for the Immulite assay platform (http://ticemed_sa.upmc.fr/sd_score/).

Quadriceps muscle biopsies were taken to assess changes in SDH activity using immunohistochemistry. The biopsies were frozen immediately after excision, mounted onto cork disks, frozen in 2-methylbutane at −196°C, and finally 12-µm sections were cut using a cryostat and mounted onto polysine (VWR) microscope slides, which were stored at −25°C until use. All samples were analyzed in a single batch. Thawed sections were incubated for 1 h at 37°C in 0.5 M Sorenson’s buffer containing 0.5 M sodium succinate and 1 mg/mL nitroblue tetrazolium. After rinsing in water, the sections were fixed in formal saline and mounted in glycergel for optical density analysis using a light microscope equipped with a Cool-Snap digital camera and Image Pro plus an image analysis software (Media Cybernetics, Wokingham, UK). Four random fields of view at 100× magnification were used from each section. Black and white images were captured, background corrected, and calibrated for incident light. An average optical density value for each was measured.

The article "Effects of Growth Hormone Replacement on Peripheral Muscle and Exercise Capacity in Severe Growth Hormone Deficiency" was published in 2018. Journal: Front Endocrinol (Lausanne).

Exercise capacity was assessed calculating the maximal oxygen consumption (VO_2_max) following cardiopulmonary exercise test, using a modified Bruce protocol. During the test, patients wore a tightly fitting facemask to which was connected a capnograph and a sample tube enabling online measurement of ventilation and metabolic gas exchange. A respiratory exchange ratio (RER) >1 was taken to suggest a maximal effort together with an attainment of at least 85% of maximal heart rate.

### Statistical Analysis

A power analysis based on the SDH could not be undertaken as there were no previous studies for reference. Therefore, change in lean body mass with rGH therapy was used as a surrogate of rGH treatment efficacy: for a significant reduction in total body fat, a sample size of eight patients in a crossover design was calculated giving 80% power to detect a mean decrease of 1.2% of total body fat, with a two-sided alpha error of 0.05 (17).

Mean changes obtained at the end of rGH treatment were compared with those at the end of the placebo phase, using the paired Student’s *t*-test. The data were normally distributed when tested with Kolmogorov–Smirnov test. Adjusting for period effect was carried out by the Hills-Armitage method (18). Statistical analysis was performed using the Stata Statistical Computer package (StataCorp, 2007). Results were considered statistically significant if the two-tailed *p* value was <0.05.

## Results

All patients completed the study and were compliant with the medication. Baseline study characteristics are included in Table 2. No significant side effects were reported other than transitory local discomfort following muscle biopsy; patients were assessed at each clinic visit.

**Table 2:** Baseline values and after 3 months placebo and 3 months recombinant growth hormone therapy.

	Baseline	Placebo (3 months)	rGH (3 months)	*p*value
**Baseline characteristics of the subjects**				
Fat mass (%)	37.4 ± 9.8	37.6 ± 10.7	36.2 ± 10.4	0.58
BMI (kg/m^2^)	33.9 ± 5.8	34.1 ± 6.18	33.9 ± 6.2	0.48
W–H ratio	0.97 ± 0.23	0.94 ± 0.07	0.93 ± 0.05	0.41
SBP (mmHg)	134 ± 14	129 ± 15	136 ± 16	0.06
DBP (mmHg)	83 ± 10.8	77 ± 8.6	79 ± 13	0.4
Glucose(mmol/L)	5.5 ± 0.7	5.1 ± 1.05	5.1 ± 0.9	0.99
HbA1c (%)	6.08 ± 1.02	5.6 ± 0.4	5.8 ± 0.8	0.12
IGF1 ug/L	115.5 ± 47	121 ± 50	189 ± 71	<0.005
T.Chol. (mmol/L)	5.5 ± 0.7	5.6 ± 0.8	5.4 ± 0.7	0.06
TG (mmol/L)	1.6 ± 1.1	1.5 ± 0.9	1.4 ± 0.7	0.09
SDH (OD units)	0.052 ± 0.03	0.073 ± 0.02	0.093 ± 0.02	<0.05
**Cardiopulmonary exercise test**				
Peak VO_2_	26.2 ± 7.6	24.3 ± 6.2	24.1 ± 7.5	0.51
VE/VCO_2_	27.6 ± 3.9	26.9 ± 4.5	28.3 ± 5.65	0.86
AT	15.4 ± 4.2	15.2 ± 4.8	15.6 ± 5.7	0.95
Peak RER	1.1 ± 0.07	1.08 ± 0.14	1.06 ± 0.14	0.06
Exercise time (s)	691 ± 267	730 ± 245	661 ± 239	0.64
Pulse at max exercise	152 ± 30	154 ± 30	147 ± 26	0.9

*AT, anaerobic threshold; BMI, body mass index; BP, systolic blood pressure; DBP, diastolic blood pressure; HbA1c, glycosylated hemoglobin; IGF1, serum insulin-like growth factor 1; OD, optical density; RER, respiratory exchange ratio; SDH, succinate dehydrogenase; T.Chol., total cholesterol; TG, triglyceride; VE/VCO_2_, slope of the relation between ventilation and carbon dioxide production; VO_2_, peak oxygen consumption; W–H ratio, waist–hip ratio*.

The article "Effects of Growth Hormone Replacement on Peripheral Muscle and Exercise Capacity in Severe Growth Hormone Deficiency" was published in 2018. Journal: Front Endocrinol (Lausanne).

### Effects on Muscle Oxidative Capacity

Succinate dehydrogenase increased significantly (*p* < 0.001) for the combined arms comparing baseline just prior to rGH therapy to 3 months rGH therapy (0.052 ± 0.030 versus 0.093 ± 0.022, *p* < 0.0001). There was a difference between placebo and rGH-treated groups (0.073 ± 0.02 versus 0.093 ± 0.02, *p* < 0.05) (Figure 2).

**Figure 2:** **(A)** Section of quadriceps muscle from a patient deficient in growth hormone at the start of the trial. Blue staining denotes the mitochondrial enzyme succinate dehydrogenase. **(B)** Section of quadriceps muscle from the same patient at the end of the trial after 3 months treatment with growth hormone. Staining as above.

### Effects on Exercise Capacity

No significant effects in peak oxygen consumption (peak VO_2_), slope of the relation between ventilation and carbon dioxide production (VE/VCO_2_), anaerobic threshold, RER, exercise time, or pulse at maximal exercise were noticeable (Table 2). There was no correlation between SDH and exercise capacity (*p* > 0.05).

### Effects on IGF1 and Cardiovascular Markers

Recombinant GH replacement normalized IGF1 levels within the reference range. The incremental difference in total body fat mass determined by Tanita measurement between active and placebo arms was calculated for each patient (placebo 0.2 ± 0.2% versus 3.2 ± 0.3% active) and was significantly reduced (*p* < 0.05). IGF1 levels did not differ with 3 months of placebo therapy and normalized with 3 months rGH therapy; these patients were then continued on growth hormone at the end of this period. For those on rGH treatment that was started on rGH (IGF1 120 ± 51 μg/L) and crossed over to placebo, IGF1 levels fell to those of pretreatment after rGH was withdrawn (123 ± 50 μg/L, *p* = 0.23) before they too were recommenced on rGH therapy at the end of the study period. No significant differences were observed in body mass index (BMI), waist–hip ratio, blood pressure, glucose, HbA1c, total cholesterol, or triglycerides (Table 2). There was no correlation between SDH and cardiovascular risk markers (*p* > 0.05). IGF1 SDS scores at baseline, 3 months active, and then 3 months placebo were −1.21 ± 0.9, 1.29 ± 0.9, and −1.07 ± 1.0, respectively, for the group that had active treatment first followed by placebo. IGF1 SDS scores at baseline, 3 months placebo, and then 3 months active were −2.2 ± 1.1, −2.1 ± 1.2, and 0.1 ± 0.8, respectively, for the group who had placebo followed by active treatment. While the baseline IFG-1 SDS scores differed at baseline, this difference was not significant (*p* < 0.06).

The article "Effects of Growth Hormone Replacement on Peripheral Muscle and Exercise Capacity in Severe Growth Hormone Deficiency" was published in 2018. Journal: Front Endocrinol (Lausanne).

## Discussion

GH either directly or *via* an IGF1-dependant action not only mediates trophic effects in the skeletal muscle promoting muscle cell proliferation, differentiation, and survival but also appears to modulate protective responses on muscles exposed to oxidative stress (19). Patients with GHD are exposed to an abnormal metabolic environment that is likely to perpetuate high levels of ROS, downregulating IGF1-1 signaling further and increasing oxidative stress and mitochondrial dysfunction. This high gradient of superoxide molecules could disrupt the individual components of the mitochondrial electron transport chain including SDH. By administering GH, one could postulate that these mitochondrial abnormalities could be ameliorated, in addition to a more direct, positive effect on body fat and lipid profile.

Our study suggests that at the end of the 3-month rGH treatment period, SDH reflective of mitochondrial oxidative activity in the peripheral muscle was higher in the rGH group compared to the placebo group that would be in accord with the reduced oxidation that was seen for rGH replacement over a 6-week period (20). However, the increased SDH activity did not reflect a significant improvement in the subject’s aerobic capacity measured by VO_2_max that have been shown to occur following prolonged rGH therapy (21, 22). In this context, similar increases in VO_2_max can be achieved either individualizing rGH dose or using higher doses based on the body weight (23–26); however, a study using a similar dose of GH replacement reported an increase in anaerobic but not aerobic (VO_2_max) after 6 months therapy (27), due to evidence that GH stimulates the anaerobic and suppresses the aerobic energy system (28). SDH is also influenced by the level of physical training, i.e., lower in subjects who lead a sedentary life compared to those who exercise (29) intermittently, continuously, or following endurance training (30, 31). Furthermore, the introduction of moderate exercise in patients with GHD can mimic the effect of GH replacement on physical activity (26). Therefore, it would have been of interest to have had placebo and rGH groups in combination with exercise to determine the effect of GH, exercise, or both on SDH, given the data that indicate that GH does not enhance muscle strength, power, or aerobic exercise capacity, but improves anaerobic exercise capacity (32). It should be noted that this was an obese population with a mean BMI greater than 30, and it is not clear if these results would be applicable to a lean population.

The article "Effects of Growth Hormone Replacement on Peripheral Muscle and Exercise Capacity in Severe Growth Hormone Deficiency" was published in 2018. Journal: Front Endocrinol (Lausanne).

The adequacy of rGH replacement in this study was shown by the normalized IGF1 levels. However, this dose and/or the length of treatment was inadequate to improve weight, central obesity, and hypercholesterolemia. It has been suggested that patients with the most adverse lipid profile benefit the most following rGH replacement (33) with changes in lipid and body composition seen between 6 months and a year (34–37) and continue up to 10 years (38) and therefore not seen in this 3-month period.

Our study has a number of limitations. This was a small study although offset by the crossover design. The duration of GH therapy was short that may have been insufficient for the full spectrum of cardiovascular benefit to have accrued. However, the effect of GH on oxidation may be seen after 6 weeks of GH replacement therapy and therefore 3 months treatment would have been sufficient for muscle mitochondrial function changes to be evident (20), and indeed this was seen. However, while IGF1 levels returned to baseline after the withdrawal of rGH, the washout period of 2 weeks may not have been sufficient between the active group changing to the placebo group so that the magnitude of the SDH changes may have been larger with a longer washout period. It should also be noted that GH therapy is influenced by gender, and to maintain the blinding of the study, there was no dose titration; therefore, the absence of dose titration could potentially influence the findings due to variability on GH responsiveness between men and women. A further limitation is that more extensive assessment of mitochondrial function with citrate synthase activity and cytochrome C oxidase activity would have been ideally performed, but this would have necessitated a larger biopsy than was taken to minimize subject discomfort.

The article "Effects of Growth Hormone Replacement on Peripheral Muscle and Exercise Capacity in Severe Growth Hormone Deficiency" was published in 2018. Journal: Front Endocrinol (Lausanne).

All the patients normalized IGF1 within reference range, but due to the study design, it was not possible to further titrate the rGH; however, normalization of IGF1 with a reduction of the body fat suggests that the patients were replaced adequately. The length of GH deficiency in the study may have been too short to have allowed more of a GH deficiency spectrum to develop after the active treatment phase.

In summary, short-term, fixed rGH for 3 months had a significant effect on mitochondrial function and favorably improved total fat mass and IGF1 levels although cardiovascular risk factors and exercise capacity did not differ over this time period.

## Ethics Statement

The study followed the declaration of Helsinki guidelines and was approved by the Hull and East Riding ethics committee. The trial registration number is ISRCTN94165486.

## Author Contributions

SG did the data analysis and wrote the manuscript. TS, ZJ, and SA revised and edited the manuscript. All authors approved the manuscript for submission.

## Conflict of Interest Statement

The authors declare that the research was conducted in the absence of any commercial or financial relationships that could be construed as a potential conflict of interest.
